The article "Analysis of the Influence of Library Information on the Utilization of Regional Environmental and Ecological Resources: From the Perspective of Intelligent Adaptive Learning" was retracted in 2023. Reasons: signs of a paper mill; unreliable results or conclusions; concerns about the data; concerns about the peer review.

# Analysis of the Influence of Library Information on the Utilization of Regional Environmental and Ecological Resources: From the Perspective of Intelligent Adaptive Learning

**DOI:** 10.1155/2022/1110105

**Published:** 2022-09-29

**Authors:** Shujie Jiang, Xuemei Yang

**Affiliations:** Nanyang Normal University, Nanyang, 473061 Henan, China

## Abstract

In order to further develop and improve the management theory of public libraries, this paper studies the impact of library information on the utilization of regional environmental resources from the perspective of intelligent adaptive learning. Firstly, based on the data envelopment analysis method, this paper measures the efficiency of Public Libraries in various regions of China. Then, using Tobit model, this paper analyzes the environmental factors affecting the efficiency of public libraries from three aspects: financial allocation, per capita GDP, and per capita years of education. The results show that there is a significant correlation between per capita GDP, per capita years of education, and the efficiency of public libraries. There is a significant negative correlation between per capita GDP and public library efficiency (the coefficient is −5.73x10^−6^, and the probability of two-sided *t*-test is 0.0229); There is a significant positive correlation between the number of years of education per capita and the efficiency of Public Libraries (the coefficient is 0.0684, and the probability of two-sided *t*-test is 0.0169). Conclusion: This study provides a reference for the performance evaluation of provincial public libraries.

## 1. Introduction

Public library is an important part of the public cultural system. It is an important institution to transmit scientific and cultural knowledge, carry out social education, and preserve human cultural heritage. It plays an important role in promoting the development of social advanced culture, popularizing social civic education, and promoting social information construction and services. In recent years, with the construction of public cultural service system covering the whole country being put on the national agenda, grass-roots libraries below the county level have been paid more and more attention by governments at all levels [1]. Compared with public libraries above the provincial level, grass-roots libraries mainly refer to district, county, street, and community libraries in cities, while in rural areas they mainly refer to county, township, and village libraries. Among them, district and county level public libraries are the public libraries with the largest number, the widest coverage and the largest number of service people, and play an irreplaceable role in the development of social economy and culture. On the other hand, with the continuous development of technology, high resource integration, and rapid resource acquisition have become the development requirements of contemporary public libraries. Therefore, the operating efficiency of libraries has attracted more and more attention [2]. Efficient libraries will certainly be able to provide more high-quality, stable, and satisfactory services, so as to give full play to their own advantages in similar libraries, while inefficient libraries will have a bad impression on readers and affect their own development. This requires us to evaluate the operation efficiency of public libraries, so as to analyze the current situation of library operation, and put forward some suggestions on its development direction. As far as the public library is concerned, it is a regional knowledge portal, providing a “lifelong learning, independent judgment, and cultural development environment” for all local people. It can be said that the public library plays a great role in the national cultural and educational system and the development process of a harmonious society. As a main form of grass-roots libraries, district and county-level libraries are the library groups closest to public life and concerned by the society and the public [3]. Compared with other libraries, the indicators and utilization of district and county-level public libraries can better reflect the social, economic, and cultural level of a region. Through the evaluation and analysis of the efficiency and influencing factors of district and county-level public libraries, it will provide theoretical and practical basis for the healthy development of library undertakings, so as to provide better services for the public. Therefore, the efficiency evaluation of district and county-level public libraries will be conducive to optimizing the resource allocation of libraries, ensuring the effective use of resources, making them better provide intellectual support for economic construction and social development, so as to create greater economic value.

## 2. Literature Review

Zhu, J. Q. and others believe that the concept of library service includes two basic aspects: quality and value. The evaluation standard of service quality is whether the library can meet the needs of users, and the service value is the service effect recognized by the fund provider. This concept has a wide influence in the early western scholars' research on library evaluation, and also laid a theoretical foundation for future research on Libraries [4]. Liu, Z. and others pointed out that any type of service evaluation can be divided into three perspectives: effect evaluation, cost effect evaluation, and cost-benefit evaluation [5]. Among them, the effect evaluation is based on the satisfaction of the service object to its use needs. Cost effectiveness evaluation is based on the relationship between the service performance level and the relevant inputs consumed to achieve this goal. Cost benefit evaluation is whether the value of service output is reasonable for the cost paid. Mansky, S. and other believe that the criteria for evaluating the quality of libraries can be fabricated, but their credibility is damaged by artificially splicing indicators. In addition, he further affirmed the two concepts of quality and value, and believed that resource input is the basis for the development of library services. Without relevant resource input, libraries will lose the basis for their existence and development. Therefore, library evaluation based on resource utilization is an important basis for reflecting the quality and value of libraries [6]. Talaat, M. and others put forward “it is useful for us to make money produce value, especially if we can prove that a small increase in money will produce a large increase in value” by introducing cost-benefit and cost-benefit theories, which shows that both from the perspective of government supervision to provide financial support for libraries and libraries themselves, we need to pay attention to the relationship between library input costs and output benefits [7]. Saif, Y. and others took the British public libraries before and after the reorganization as the object, put forward the relevant assumption that the service efficiency of public libraries will change over time, compared the efficiency of British public libraries before and after the reorganization, and evaluated the reorganization effect of libraries [8]. Olney, A. M. and others used DEA model to analyze the efficiency of 118 University Libraries in 6 countries, and ranked the efficiency of university libraries by comparing the efficiency values among university libraries [9]. Balachandran, P. V. used DEA model to evaluate the resource utilization efficiency of University Libraries. Through analysis, they concluded that the use degree of electronic resources has a significant impact on library efficiency, so it is necessary to strengthen the digital construction of University Libraries [10]. Karthikeyan, L. and others used a two-stage DEA model to evaluate the efficiency of American public libraries, evaluated the impact of intermediate output on efficiency in terms of services and project results, and estimated the optimal level of nonperforming loan ratio to promote the improvement of the second stage efficiency [11].

This paper takes 31 provincial regions in China as the research object, based on the reasonable selection of input-output indicators, measures the operation efficiency of Public Libraries in different regions based on DEA method, uses Tobit regression method, and makes efficiency analysis through SE-SBM model, and discusses the environmental factors affecting the efficiency of regional public libraries.

## 3. Research Methods

### 3.1. Learning Support System

The research on the adaptive learning support system includes: intelligent network teaching system, adaptive hypermedia system, adaptive intelligent agent system, adaptive distance learning support system, semantic web adaptive learning system, two-way adaptation mechanism, etc. Module components in the system mainly include domain model, user model, adaptive model, interface module, etc. The learning support system proposed in this paper takes the learning behavior evaluation model as the center, including modules such as learner portrait and resource recommendation [12]. The structure is shown in Figure 1:

#### 3.1.1. Data Acquisition

Adaptive learning is based on data acquisition and data mining of historical data generated in the whole process of learners' learning. Therefore, libraries are required to fully perceive the learning environment, application equipment, learners' information, and other situational information. The data to be collected can be divided into basic education data, online learning data, library use data, and library behavior data. Among them, basic education data include learners' names, gender, age, student number, departments, grades, research projects, research results, etc. Online learning data includes online time, login habits, number of resource visits, link dwell time, hit rate of heat map, correct rate of exercises, assessment results, etc. Library usage data includes borrowing and returning data, portal access data, digital resource search, and download data. Library behavior data includes access control data, track tracking data, learning efficiency data, learning emotion data, etc. In terms of data acquisition methods, basic education data, online learning data, and library use data can be obtained from the corresponding databases or logs. Learners' behavior data in the library needs to be collected through devices [13, 14]. Learners' time in the library and habits of entering the library can be collected through the access control system. The trajectory of activities in the museum space can be tracked by face capture surveillance cameras and other equipment. The web browsing data of the public computer in the library can be collected by eye tracker. The writing data in the library can be collected by dot matrix digital pen. The learning emotion data in the self-study area in the library can be collected by the face capture surveillance camera. Libraries should pay attention to the legality, legitimacy, and necessity of collecting and using learners' personal data in accordance with relevant national laws and regulations [15]. All personal data shall not be provided externally, collected beyond the scope, and sensitive information shall not be publicly disclosed. Libraries should sign confidentiality agreements with cooperative units that have access to personal information and data, limit the number of contacts, establish accountability systems, and ensure data security.

### 3.2. Research Methods and Data Description

#### 3.2.1. DEA-Obit Two-Step Method

DEA method was proposed by James, Cooper, and Rhode in 1978 to evaluate the relative effectiveness of decision-making units under the “multi-input and multi-output” mode. This paper uses the CCR model of DEA method to measure the efficiency of public libraries with the national inter provincial region as the basic decision-making unit. For any decision-making unit, the CCR model in dual form can be expressed as the following formula (1):

(1) $$\begin{array}{c} {\text{M}}_{\theta ,\lambda }\text{in}\left[\theta -\varepsilon \left({\text{e}}^{\text{t}}{\text{s}}^{-}+{\text{e}}^{\text{t}}{\text{s}}^{+}\right)\right]\\ \text{S}.\text{T}.\left\{\begin{array}{c} \overset{\text{n}}{\underset{\text{i}=1}{\sum }}\lambda_{\text{i}}{\text{y}}_{\text{ir}}-{\text{s}}_{\text{s}}^{+}={\text{y}}_{0_{\text{r}}}\\ \overset{n}{\underset{\text{i}=1}{\sum }}\lambda_{\text{i}}{\text{x}}_{\text{ij}}+{\text{s}}^{-}=\theta_{{\text{x}}_{\text{j}}}\\ \lambda_{\text{i}}⩾0;\text{s}⩾0;\text{s}⩾0\\ \text{i}=1,2,\cdots ,\text{n};\text{j}=1,2,\cdots ,\text{m};\text{r}=1,2,\cdots ,\text{s} \end{array}\right., \end{array}$$

where *n* is the number of decision-making units, *m* and *s* are the number of input and output variables, respectively, x_ij_(j = 1, 2, ⋯, m) is the input element, y_ij_(j = 1, 2, ⋯, m) is the output element, and *θ* is the effective value of decision-making unit *DMU*_0_. If *θ* = 1 and s^+^ = s^−^ ≠ 0, DEA of decision-making unit is valid. If *θ* = 1 and s^+^ ≠ 0 or s^−^ ≠ 0, the decision-making unit is weak DEA effectiv. If *θ* < 1, the decision-making unit is not DEA effective.

In order to further analyze which environmental factors affect the evaluation efficiency value and their influence degree, a method called “two-stage method” is derived from DEA analysis. The first step is to evaluate the efficiency value of the decision-making unit through DEA model. The second step is to do the regression of efficiency value (dependent variable) to various environmental factors, and judge the influence direction and intensity of environmental factors on efficiency value from the coefficient of independent variable [16]. However, the efficiency value (independent variable) determined by the DEA model is limited to 0 and 1. If the model is directly regressed by the ordinary least square method, the parameter estimation will be biased towards 0. Censored regression model (also known as “Tobit model”) can solve this kind of problem, as shown in formula (2):

(2) $$\begin{array}{c} \left\{\begin{array}{c} {\text{y}}^{*}=\beta_{{\text{x}}_{\text{i}}}+\varepsilon \\ {\text{y}}_{\text{i}}={\text{y}}_{\text{i}}^{*},\text{if }{\text{y}}_{\text{i}}^{*}>0\\ {\text{y}}_{\text{i}}=0,\text{if }{\text{y}}_{\text{i}}⩽0 \end{array}\right., \end{array}$$

where *ε*_i_ ~ **N**(0, *σ*^2^), *β* is the regression parameter vector, x_i_ is the independent variable vector, y_i_^∗^ is the dependent variable vector, and y_i_ is the efficiency value vector.

Using DEA-Tobit two-step method to analyze efficiency and its influencing factors has been relatively mature in various fields. DEA-Tobit two-step method has been relatively mature in terms of method, which is worthy of reference.

#### 3.2.2. Data Source and Variable Description

Based on the existing literature on library performance evaluation and the availability of data, this paper selects 31 provinces and cities in Chinese Mainland as the spatial decision-making unit (DMU) for the measurement and evaluation of input-output efficiency of public libraries. The input variables include five aspects: the number of Public Libraries (number), the number of employees (number), the total collection of books (thousands of books, pieces, and sets), the construction area of public houses (thousands of square meters), and the number of seats in reading rooms (thousands). The output variables include the cumulative number of valid library cards issued (1000), the total circulation of people (1000), and the number of books and documents borrowed (1000). All data are from the China Library Yearbook.

When using DEA method to evaluate efficiency, we need to meet the principle of “isotropy”, that is, there must be a strong positive correlation between input and output variables, so as to ensure that increasing an input will not reduce an output instead. The commonly used method is to detect it by Pearson correlation test. The calculation results of SPSS17.0 are shown in Table 1:

It can be seen from Table 1 that the correlation coefficients between input variables and output variables in all provinces and cities are positive, and can pass the two-tailed test at the significance level of 10% or 1%, which shows that the input-output index meets the principle of “homogeneity” required by the model and is reasonable.

The focus of this paper is to determine the environmental factors affecting the efficiency of regional public libraries, which has not been considered in the existing literature. Given the constraints of resource conditions, different external environments may have an important impact on the efficiency of public libraries. Generally speaking, the government's attention to public libraries, the level of local economic development, and the education level of local residents may be the factors affecting the efficiency of public libraries. This paper also discusses the impact of the external environment on the efficiency of public libraries from three aspects. Among them, the government's emphasis on public libraries is described by the financial allocation (1000 yuan) variable, and the economic development level of various regions is measured by per capita GDP. As for the education level of residents, considering the availability of data, it is measured by the number of years of education per capita in each region [17, 18]. Because the “China Statistical Yearbook” gives the sampling data of the population aged 6 and above in various regions who have not attended school, primary school, junior high school, senior high school, and junior college or above. According to the weighted average of the five types of population, the time of education is 0, 5, 8, 11, and 14.5 years, respectively, from which the average years of education of the local population can be calculated. The financial allocation data are from the China Library Yearbook, and the per capita GDP and per capita years of education in various regions are from the China Statistical Yearbook.

### 3.3. Efficiency Analysis Based on SE-SBM Model

#### 3.3.1. Index Construction

*(1) Selection Principle*. In order to better select the evaluation indicators of service efficiency, we must grasp the selection principles of evaluation indicators in order to make the evaluation results scientific and reasonable. This paper takes SMART, a principle commonly used in performance research, as the basic principle of index selection: (1) The principle of specificity. (2) Measurable principle. (3) Realizable principle. (4) The principle of relevance. (5) Time bound principle. To sum up, this paper selects appropriate variable data from five perspectives: clarity, measurability, realizability, relevance, and timeliness.

*(2) Selection Basis*. From the existing research, it can be seen that domestic and foreign scholars choose input indicators from three aspects: human, material, and financial resources, and output indicators from the flow of people, the number of books borrowed, or the volume of business, but there are still some differences in details. For example, some scholars tend to use the total value, and some scholars tend to choose the average value. Therefore, we need to combine the actual situation of the current research object to determine the evaluation index.

*(3) Determination of Indicators*. The primary function of the public library is to provide literature borrowing, information consulting, and information retrieval services for the public in the service area. Therefore, the selected indicators need to directly reflect the service function of the public library. In terms of the selection of investment indicators, the number of books collected, the number of employees, the opening hours of the library, the number of reading rooms, the purchase funds of new books, the total investment of funds, the area of the library, and other indicators reflect the resource investment of the public library. The circulation person times, the number of books borrowed, the number of valid library cards issued, and the business volume reflect the service volume of the public library services to the public [19].

In terms of investment indicators, the construction of public libraries is inseparable from the investment of human, material, and financial resources. From the perspective of manpower, the number of employees represents the infrastructure of human services. The site management, activity development, borrowing, and consulting of the library must be completed with the participation of service personnel. Public libraries without manpower will lose their due service functions. From the perspective of material resources, the buildings of the public library provide the necessary space for services, and are the space carrier for the realization of public library services, and the housing area is an important indicator to measure the space carrying capacity. In addition, the most important and core product of the public library is its collection of books and documents. Only through the collection can its functions of information dissemination, browsing, and borrowing be realized. Therefore, the number of books collected is also an important basis for public library service investment. From the perspective of financial resources, the expenditure reflects the necessary expenditure to support the operation of the whole venue. The purchase of new books, the holding of activities, the maintenance of venues, the renewal of equipment, and so on are inseparable from the support of relevant funds.

In terms of output indicators, unlike the private sector, public libraries do not take business income and operating profit as the basis for measuring service results. In essence, they want to provide public services for the public. Therefore, the most intuitive statistical method is to use the total circulation and book lending times that can best reflect the output results. Among them, the total circulation person times reflect the degree to which the public go to the public library to participate in the service, and the number of books and periodicals borrowed reflects the degree to which the public use the cultural products of the public library [20].

To sum up, this paper selects the expenditure, the number of books collected, the public area of houses, and the number of employees in terms of input indicators, and selects the total circulation person times and book lending times in terms of output indicators, as shown in Tables 2–5 below.

## 4. Result Analysis

### 4.1. DEA Efficiency Analysis

DEA method has two modes: input-oriented and output-oriented. Input-oriented mode refers to the appropriate adjustment and control of input under the premise of fixed output, while output-oriented mode refers to the adjustment and control of output under the premise of fixed input [21]. In the operation of public libraries, the input-output ratio is easy to control. Therefore, this paper selects the input-oriented DEA model for analysis. Using DEAP2.1 software package to calculate the efficiency value of Public Libraries in various provinces and regions in China. The calculation results are shown in Table 6, Figures 2–4.

It can be seen from Table 4 and Figures 2–4 that the regions at the forefront of efficiency include 14 provinces and cities, including Beijing, Inner Mongolia, Shanghai, Fujian, Jiangxi, Guangdong, Guangxi, Hainan, Chongqing, Guizhou, Yunnan, Gansu, Qinghai, and Ningxia, accounting for 45.2% of all regions. These 14 provinces and cities are both technically efficient and scale efficient. Based on the current input scale, the output has reached the optimal level. Unless the input is partially or completely increased, or a certain amount of output is reduced, its output cannot be increased under the existing technical level. The pure technical efficiency and scale efficiency of DEA noneffective units are investigated, respectively. The calculation results show that Hebei, Shanxi, Liaoning, Jiangsu, Anhui, Henan, Hubei, Hunan, Sichuan, Tibet, Shaanxi, and Xinjiang are pure technical efficiency rather than scale efficiency, accounting for 38.7% of all regions. According to the current output, the input of these regions can not be reduced. The remaining five provinces and cities of Tianjin, Jilin, Heilongjiang, Zhejiang, and Shandong are neither technically effective nor scale effective, indicating that even if some of their inputs are reduced, it is possible to maintain the current output level.

#### 4.1.1. Analysis of Environmental Impact Factors

DEA analysis results show that the efficiency of Public Libraries in various regions of China is inconsistent. As mentioned above, the factors affecting the efficiency of public libraries include the importance the government attaches to public libraries, the level of economic development in various regions, and the education level of residents in various regions. Next, Tobit regression is carried out with the technical efficiency of Public Libraries in various regions as the dependent variable and the financial allocation, per capita GDP and per capita years of education in various regions as the independent variables. The model is constructed as follows:

(3) $$\begin{array}{c} \text{TEF}=\alpha_{0}+\alpha_{1}\text{FIN}+\alpha_{2}\text{PGDP}+\alpha_{3}\text{EDU}+\varepsilon_{\text{i}}. \end{array}$$

Among them, TEF represents the technical efficiency of the public library, FIN represents the financial allocation, PGDP represents the per capita GDP, EDU represents the per capita years of education, *α*_0_, *α*_1_, *α*_2_, *α*_3_ are the coefficients to be estimated in the model, and *ε*_i_ is the random disturbance term. The estimated results of software eviews6.0 are shown in Tables 7 and 8.

The estimated results in Tables 7 and 8 shows that there is a significant correlation between per capita GDP, per capita years of education, and the efficiency of public libraries. There is a significant negative correlation between per capita GDP and public library efficiency (the coefficient is −5.73x10^−6^, and the probability of two-sided *t*-test is 0.0229). There is a significant positive correlation between the number of years of education per capita and the efficiency of Public Libraries (the coefficient is 0.0684, and the probability of two-sided *t*-test is 0.0169). The number of years of education per capita is significantly positively correlated with the efficiency of public libraries, that is, the more developed education is, the higher the efficiency of public libraries is. This fully shows that there is a close relationship between the operation of public libraries and the education level of readers. Readers with higher education tend to go to the library to seek literature resources, so as to promote the more effective use of public library resources, and then improve the efficiency of public libraries.

The negative correlation between per capita GDP and public library efficiency seems to be contrary to common sense. Generally speaking, the material and cultural needs of the public in economically developed areas should be higher, so as to play a positive guiding role in the operation of public libraries, and then improve the efficiency of public libraries. However, this empirical study does not support this conclusion. In-depth analysis is not difficult to explain, in economically developed areas, readers often have higher demand. However, the decision-making of Public Libraries in China is dominated by administration, and the decision-makers directly affect the resource supply of public libraries. When the interests of decision-makers are inconsistent with or even contrary to the needs of readers, it is easy to see the phenomenon of supply exceeding demand, which makes the library resource supply appear structural imbalance. In this way, the resource allocation of Public Libraries in economically developed areas is difficult to match the higher needs of readers, resulting in lower efficiency.

Financial allocation is positively related to the efficiency of public libraries, but the impact is not significant, which shows that financial allocation does play a positive role in promoting the efficiency of public libraries, but from the national level, this effect is not obvious [22]. This conclusion further confirms the low efficiency of the use of funds in public libraries in China, and the financial allocation has not effectively improved the efficiency of public libraries. The reasons may be as follows: first, the service object of the public library are the readers, but it is difficult to grasp the needs of readers, which makes it difficult for funds to allocate resources effectively, resulting in the failure of financial allocation to improve the efficiency of the public library. The second may be that the limited funds are seriously disconnected from the needs of readers when allocating resources, such as building large-scale venues in areas with small reader needs, colluding with booksellers to purchase a large number of overstocked books, etc.

Remove the variable financial allocation in model 1 that has no significant relationship with the efficiency of public libraries, and observe the change of regression results. See model 2 for the results. The impact of variables in model 2 on the efficiency of public libraries is still significant, and the coefficient symbols are consistent with the original model. Therefore, it can be considered that the impact of these variables on the efficiency of public libraries are stable and reliable.

### 4.2. Data Analysis of SE-SBM Model in a City

This paper selects the SE-SBM-I-V model in the SE-SBM model, and the statistical tool is MaxDEA. The assumption of the model is that when the output is fixed, the input is nonradial and the return to scale is variable, that is, the input and output of the decision-making unit can be changed in different proportions. Taking the relaxation variable into the consideration of the model helps to distinguish the efficiency value under the same proportion of input and output changes, and it is convenient to sort the research results.

#### 4.2.1. Pure Technical Efficiency

Pure technical efficiency score (VRS) reflects the production efficiency of each input factor of the decision-making unit at the optimal production scale. Its efficiency value is affected by the technology and management of the decision-making unit, and it is the efficiency of resource utilization level after excluding the impact of changes in return to scale.

As shown in Table 9 below, from 1999 to 2018, the pure technical efficiency of a city's public library showed a trend of decreasing first and then increasing. Among them, the efficiency values in 1999, 2000, 2001, 2003, 2012, 2016, 2017, and 2018 were higher than 1, indicating that the pure technical efficiency in the above years was relatively effective excluding the impact of scale changes. Therefore, the technical and management resources of a city's Public Library in these years were better utilized. While the technical efficiency value in other years is less than 1, indicating that the technical efficiency is insufficient and the resources invested in technology and management have not been fully used.

To form effective output. As shown in Figure 5 below, from the change of pure technical efficiency, it can be divided into two stages: from 1999 to 2010, except for 2003 and 2008, the pure technical efficiency showed a significant downward trend, and decreased year by year. 2010 was the minimum efficiency, and the efficiency value was 0.297, indicating that during this period, the resource utilization and service output level of a municipal public library were declining. From 2011 to 2018, the pure technical efficiency began to reverse the downward trend and rebounded. In particular, 2012 was the maximum efficiency value, and the efficiency value was 1.265. The efficiency value of the previous three years was less than 1 from 2013 to 2015, which was relatively invalid, while the efficiency value from 2016 to 2018 was higher than 1, which was relatively effective. The efficiency value in 2017 was the maximum efficiency value, and the efficiency value was 1.497. It shows that from the perspective of technology and management, a municipal public library has performed well in the level of resource utilization and service output in these three years, and the efficiency value has been greatly improved compared with that before 2010.

#### 4.2.2. Comprehensive Technical Efficiency

Technical efficiency score (CRS) is the product of pure technical efficiency and scale efficiency. Different from pure technical efficiency, the comprehensive technical efficiency considers the impact of changes in production scale on the resource utilization of decision-making units. The calculation result is the efficiency under the condition of constant scale, which is a comprehensive evaluation of the resource allocation capacity of decision-making units. As shown in Figure 6 below, overall, the comprehensive technical efficiency value from 1999 to 2018 also showed a trend of first decreasing and then increasing. Among them, the efficiency value in 1999, 2000, 2003, 2012, 2017, and 2018 is greater than 1, which is relatively effective, indicating that under the condition of comprehensively considering the changes in the size of the library, the resource utilization and service output of the public library are better, while the efficiency in other years is less than 1, which indicates that the resources invested in these years have not formed effective output.

From the perspective of the change of comprehensive technical efficiency, it can also be divided into two stages: from 1999 to 2010, except for 2003 and 2008, the comprehensive technical efficiency showed a downward trend, and in 2010, it reached the minimum efficiency value, with the efficiency value of 0.285. Since 2011, the downward trend of efficiency value has changed, and there has been an upward trend. Among them, 2012 is the maximum efficiency value, and the efficiency value is 1.228, while the comprehensive technical efficiency from 2013 to 2016 fell back to a lower level. The efficiency value less than 1 is relatively ineffective, only slightly higher than the efficiency in 2009 and 2010, and the growth change range is small. It shows that the comprehensive capacity of resource allocation of a municipal public library during these four years is insufficient, and no good output has been formed. The efficiency value in 2017 and 2018 is higher than 1, and 2017 is the maximum efficiency value, and the efficiency value of 1.482 is relatively effective, reflecting that the level of resource utilization and service output in this year is the best year since the research year.

#### 4.2.3. Scale Efficiency

Scale effect score (SE) is the ratio of comprehensive technical efficiency to pure technical efficiency. It represents the ratio of the actual production scale to the optimal production scale. The value range is 0 to 1. The larger the value, the closer the actual production scale is to the optimal production scale.

As shown in Figure 7 below, the change of scale efficiency from 1999 to 2018 is different from that of pure technical efficiency and comprehensive technical efficiency. The scale efficiency from 1999 to 2012 is between 0.88 and 1 except for 2003, which indicates that the overall production scale of a city's Public Library in these years is close to the optimal. From 2013 to 2016, the scale efficiency decreased significantly. In particular, the scale efficiency in 2016 was 0.310, which was the minimum value of scale efficiency. Combined with the pure technical efficiency value of 1.162 and the comprehensive end efficiency value of 0.360 in that year, it can be found that although a municipal public library achieved relative efficiency in technology and management in 2016, there was a gap between the actual production scale and the optimal production scale. Therefore, the service output of public libraries is limited from the scale, resulting in the relatively ineffective comprehensive technical efficiency in that year. The scale efficiency in 2017 and 2018 is close to 1, indicating that a municipal public library has expanded its scale in these two years, making the actual production scale tend to the best scale, so the comprehensive technical efficiency is relatively effective.

#### 4.2.4. Return to Scale

Returns to scale (RTS) refers to the output change caused by the change of various production factors in the decision-making unit in the same proportion under other conditions unchanged. It reflects the proportional relationship between the change of production scale and the resulting output change.

In the past 20 years, returns to scale have increased in all years except 2003, 2011, and 2015. This reflects that the year of increasing returns to scale increases with the level of scale, and the growth rate of output income is higher than that of resource input, which has obvious characteristics of economies of scale. With the expansion of production scale in 2003, 2011, and 2015, the growth rate of output and income of a city's public library did not keep up with the growth level of resource input, indicating that the relevant inputs used for library construction were not translated into service output in time, and the utilization level of unit production factors failed to adapt to the changes in scale.

## 5. Conclusion

This paper uses DEA obit model to measure the efficiency of China's provincial public libraries, and analyzes its environmental factors. The results of DEA analysis show that at present, only 45.2% of provinces and cities in China are at the forefront of efficiency. The following Tobit model analysis explains the impact of the external environment on the efficiency of public libraries from three aspects: financial allocation, per capita GDP, and per capita years of education in various regions, and draws some relevant conclusions. There are still some areas that need to be improved in this paper. First of all, this paper only explains the three factors that affect the efficiency of public libraries. Whether there are other factors and how to affect them are not considered due to the unavailability of data. Secondly, the empirical analysis of this paper shows that the per capita GDP and the per capita years of education in various regions have a significant impact on the efficiency of public libraries, and these two factors are not excluded in the efficiency evaluation. Then, after excluding environmental factors, will the efficiency of Public Libraries in various regions change? This is also the research content that the author will consider soon. Finally, this paper mainly studies the horizontal comparison of the efficiency of Public Libraries in various regions, but does not involve vertical changes. Subsequent research will consider this issue.

## Figures and Tables

**Figure 1:** Structure diagram of adaptive learning system.

**Figure 2:** DEA technical efficiency values of Public Libraries in various regions.

**Figure 3:** DEA pure technical efficiency value of Public Libraries in various regions.

**Figure 4:** DEA scale efficiency value of Public Libraries in various regions.

**Figure 5:** Pure technical efficiency change curve.

**Figure 6:** Change curve of comprehensive technical efficiency.

**Figure 7:** Change curve of scale efficiency.

**Table 1:** Pearson correlation coefficient of input variables and output variables.

Input item	Output item				
	Number of public libraries	Number of employees	Total book collection	Building area of public buildings	Number of reading rooms
Number of valid library cards	0.349^∗^(0.054)	0.766^∗∗∗^(0.000)	0.677^∗∗∗^(0.000)	0.914^∗∗∗^(0.000)	0.878^∗∗∗^(0.000)
Total circulation person times	0.333^∗^(0.067)	0.738^∗∗∗^(0.000)	0.666^∗∗∗^(0.000)	0.922^∗∗∗^(0.000)	0.867^∗∗∗^(0.000)
Lending times of books and documents	0.348^∗^(0.055)	0.793^∗∗∗^(0.000)	0.723^∗∗∗^(0.000)	0.955^∗∗∗^(0.000)	0.900^∗∗∗^(0.000)

**Table 2:** Input indicators for service efficiency evaluation of a public library in a city.

Secondary indicators	Data sources
Expenditure (yuan)	Statistical yearbook of a city 1999-2018
Public housing area (m2)	
Number of books collected (volume)	

**Table 3:** Output indicators of service efficiency evaluation of a public library in a city.

Secondary indicators	Data sources
Number of employees (number)	Statistical yearbook of a city 1999-2018

**Table 4:** Evaluation index of service efficiency of Public Library in a city.

Secondary indicators	Data sources
Total circulation person time (person time)	Statistical yearbook of a city 1999-2018

**Table 5:** Input and output data of Public Libraries under the jurisdiction of a city.

Particular year	Input index				Output indicators	
	Number of books collected (book)	Public area of the house (m2)	Expenditure (yuan)	Number of employees (number)	Total circulation person time (person time)	Book lending times (book times)
1999	3270000	58602	5146000	324	744000	799000
2000	3320000	40631	6818000	316	877000	723000
2001	3461000	55922	7940000	304	673000	770000
2002	3415000	55942	10820000	306	879000	906000
2003	3439000	66482	11760000	295	1253000	1242000
2004	3499000	56303	13250000	294	960000	931000
2005	3650400	55556	14905000	290	964000	1057000
2006	3770600	55195	18926000	286	1034200	1085500
2007	3904700	54592	25256000	279	1117100	819400
2008	4059000	55051	24826000	279	1453500	1171600
2009	4244000	57891	30806000	288	1078200	936700
2010	4396200	57891	34412000	287	1097200	950300
2011	4170600	55662	38361000	289	1506300	950500
2012	4656900	58025	44593000	305	2836600	1204300
2013	4937400	58558	54059000	298	1754400	1132300
2014	5069400	59558	67764000	290	1850700	1215700
2015	5228400	59558	97343000	289	1869400	1358300
2016	1689700	34096	31927000	142	773920	731380
2017	2134500	43274	36152000	132	1244900	3493800
2018	2240600	43412	33889300	137	1333600	1280500

**Table 6:** DEA efficiency values of Public Libraries in various regions.

Region	Technical efficiency	Pure technical efficiency	Scale efficiency
Average	0.936	0.982	0.953

**Table 7:** Analysis of influencing factors of public library efficiency (Model 1).

Variable	Model 1
*α*_0_	0.5456(0.0025)^∗∗∗^
*α*_1_	4.07 × 10^−7^ (0.2033)
*α*_2_	−5.73 × 10^−6^(0.0229)^∗∗^
*α*_3_	0.0684(0.0169)^∗∗^
F value	2.5165(0.0793)^∗^
AdjR-quared	0.2185

**Table 8:** Analysis of influencing factors of public library efficiency (Model 2).

Variable	Model 2
*α*_0_	0.5691(0.0018)^∗∗∗^
*α*_2_	—3.76 × 10—6(0.0522)^∗^
*α*_3_	0.0634(0.0256)^∗∗^
F value	2.8536(0.0745)^∗^
AdjR-quared	0.1693

**Table 9:** Efficiency value results calculated by SE-SBM model.

Particular year	Comprehensive technical efficiency (CRS)	Pure technical efficiency (VRS)	Scale efficiency (SE)	Return to scale (RTS)
1999	1 .116	1.122	0.995	Increment (+)
2000	1.082	1.126	0.961	Increment (+)
2001	0.632	1.001	0.632	Increment (+)
2002	0.692	0. 785	0.881	Increment (+)
2003	1.116	1 .124	0.992	Decrement (-)
2004	0.655	0.73	0.896	Increment (+)
2005	0.644	0.718	0.897	Increment (+)
2006	0.568	0. 617	0.922	Increment (+)
2007	0. 375	0. 395	0.95	Increment (+)
2008	0. 668	0. 673	0.992	Increment (+)
2009	0. 299	0.335	0. 892	Increment (+)
2010	0. 285	0.297	0. 960	Increment (+)
2011	0. 339	0. 346	0. 977	Decrement (-)
2012	1 .228	1 .265	0.971	Decrement (-)
2013	0. 314	0. 402	0.781	Decrement (-)
2014	0. 328	0. 427	0.768	Decrement (-)
2015	0.334	0.433	0.771	Decrement (-)
2016	0.36	1.162	0.31	Increment (+)
2017	1.482	1.497	0.99	Increment (+)
2018	1.01	1.035	0.976	Increment (+)

## Data Availability

The labeled data set used to support the findings of this study is available from the corresponding author upon request.
